# Aldehyde Dehydrogenase Isoform 1 Predicts a Poor Prognosis of Acute Cerebral Infarction

**DOI:** 10.1155/2022/8199917

**Published:** 2022-07-15

**Authors:** Jing Yang, Jie Duan, Meifang Li, Haidong Sun, Yongsheng Sun, Wei Pan, Haixiang Xi

**Affiliations:** ^1^Department of Encephalopathy, Wuhan Hospital of Traditional Chinese Medicine, Wuhan, China; ^2^Department of Orthopedics, Wuhan Hospital of Traditional Chinese Medicine, Wuhan, China

## Abstract

To investigate the prognostic potential of serum aldehyde dehydrogenase isoform 1 (ALDH1) level in acute cerebral infarction, and the molecular mechanism in mediating neurological deficits, a total of 120 acute cerebral infarction cases within 72 h of onset were retrospectively analyzed. Serum ALDH1 level in them was detected by qRT-PCR. Receiver operating characteristic (ROC) and Kaplan–Meier curves were depicted for assessing the diagnostic and prognostic potentials of ALDH1 in acute cerebral infarction, respectively. An *in vivo* acute cerebral infarction model in rats was established by performing MCAO, followed by evaluation of neurological deficits using mNSS and detection of relative levels of ALDH1, Smad2, Smad4, and p21 in rat brain tissues. Pearson's correlation test was carried out to verify the correlation between ALDH1 and mNSS and relative levels of Smad2, Smad4, and p21. Serum ALDH1 level increased in acute cerebral infarction patients. A high level of ALDH1 predicted a poor prognosis of acute cerebral infarction patients. In addition, ALDH1 was sensitive and specific in distinguishing acute cerebral infarction cases, presenting a certain diagnostic potential. mNSS was remarkably higher in acute cerebral infarction rats than that of controls. Compared with sham operation group, relative levels of ALDH1, Smad2, and Smad4 were higher in brain tissues of modeling rats, whilst p21 level was lower. ALDH1 level in brain tissues of modeling rats was positively correlated to mNSS, and mRNA levels of Smad2 and Smad4, but negatively correlated to p21 level. Serum ALDH1 level is a promising prognostic and diagnostic factor of acute cerebral infarction, which is correlated to 90-day mortality. Increased level of ALDH1 in the brain of cerebral infarction rats is closely linked to neurological function, which is associated with the small mothers against decapentaplegic (Smad) signaling and p21.

## 1. Introduction

Cerebrovascular diseases have become the number one killer in China [1]. Owing to the high incidence, mortality, and recurrence, cerebrovascular diseases have brought a heavy burden to the society and families. Ischemic cerebral infarction cases account for about 70–80% of strokes, which is caused by the interruption of local cerebral blood perfusion due to cerebrovascular occlusion. Cerebral ischemia and hypoxia further result in ischemic necrosis of corresponding brain regions [2]. Neurological deficits and repair mechanisms are dynamically processed right after cerebral infarction, in which angiogenesis, destruction of the blood-brain barrier, and inflammatory response are closely interacted with each other [3]. They synergistically affect the survivals of neurons, nerve synapse repair, and regeneration, which are important for the prognosis of cerebral infarction patients.

A fast and accurate diagnosis of cerebral infarction contributes to timely treatment and satisfactory clinical outcomes. At present, CT and MRI are widely used for the diagnosis of cerebral infarction, although they have disadvantages of complicated procedures, expensive medical cost, and the demand for moving patients. It is necessary to search for noninvasive serum biomarkers that are effective in diagnosing and predicting the progression of cerebral infarction [4, 5].

ALDH1 is a member of the acetaldehyde dehydrogenase gene superfamily, which mainly catalyzes the irreversible oxidation of retinal to retinoic acid. It participates in tissue differentiation and early differentiation of stem cells [6]. In 2007, Ginestier et al. [7] initially proposed the application of ALDH1 in the research field of breast cancer stem cells. The cancer-associated function of ALDH1 in other types of cancers has emerged later [8–10]. Nevertheless, the potential function of ALDH1 in acute cerebral infarction is largely unknown. This study intends to investigate its clinical significance in predicting the prognosis of acute cerebral infarction and the underlying mechanism.

## 2. Materials and Methods

### 2.1. Subjects

Seventy acute cerebral infarction patients treated in Wuhan Hospital of Traditional Chinese Medicine were recruited. Inclusion criteria were as follows: (1) cerebral infarction was diagnosed based on the *Report of the WHO Task Force on Stroke and other Cerebrovascular Disorders* [11]; (2) cerebral infarction was confirmed by cranial CT or MRI; (3) onset of cerebral infarction ≤72 h; (4) age >18 years. Exclusion criteria were as follows: (1) intracranial hemorrhage; (2) a history of infection within 2 weeks before onset; (3) a history of malignant tumors; (4) a recent medication of hormones or immunosuppressants. Modified Rankin scale (mRS) was used for evaluating the recovery of neurological function after stroke (>2, poor prognosis; ≤2, good prognosis) [12]. Survival and adverse events were recorded. Recruited patients were followed up for 90 days. Seventy healthy volunteers receiving physical examinations in the same period, who were confirmed without stroke by cranial MRI, were included as controls. This experiment was approved by the Medical Ethics Committee of Wuhan Hospital of Traditional Chinese Medicine. Signed written informed consents were obtained from the participants before this study.

### 2.2. Blood Sample Collection and Processing

Venous blood (4 mL) was collected from every participant in the morning after overnight fast and placed in a 5 mL Eppendorf (EP) tube. The blood sample was centrifuged at 2500 g/min for 12 min, and the serum was isolated, labeled, and stored at −80°C.

### 2.3. MCAO Model

This study was approved by the Animal Ethics Committee of Wuhan Hospital of Traditional Chinese Medicine Animal Center. Sixty male Sprague-Dawley (SD) rats in the clean level weighing 230–250 g were housed in a temperature-controlled room (21 ± 2°C) on a 12: 12-h light/dark cycle (lights on at 06: 00). All rats had free access to water and food. Rats were randomly assigned to cerebral infarction group (*n* = 20), sham operation group (*n* = 20), and control group (*n* = 20). An *in vivo* acute cerebral infarction model in rats was established by performing middle cerebral artery occlusion (MCAO) [13]. Briefly, rats were anesthetized and placed in a supine position. After creating a midline incision on the neck, the right common carotid artery (CCA), external carotid artery (ECA), and internal carotid artery (ICA) were isolated. The distal end of ECA was ligated, and artery clamps were placed at the distal end of ICA and the proximal end of CCA. ECA ligation was then cut, and the artery clamp at ICA was withdrawn. A nylon suture was inserted in ECA through the opening of ECA ligation until blocking the middle cerebral artery blood flow. The suture was fixed, which was withdrawn 2 h later. Rats in the sham operation group were operated on by artery isolation, and then, the incision was sutured layer by layer. The quality of the MCAO model was evaluated by the Zea Longa score on a 5-point scale as follows: 0, absence of neurological deficits; 1, unable to fully lift the opposite forepaw; 2, circling to the opposite side; 3, falling to the opposite side; 4, unable to spontaneously walk and loss of consciousness. After anesthesia awareness, rats with 1–3 Zea Longa scores were considered as qualified modeling animals. After evaluation of neurological deficits, rats were anesthetized and sacrificed for collecting brain tissues.

### 2.4. Evaluation of Neurological Deficits

Neurological deficits of postoperative rats were evaluated using the modified neurological severity score (mNSS) at indicated time points, including tests of balance, walking, abnormal movement, sensory, reflex, and raising by tail [14]. With a range of 1–18 grades, neurological deficits were categorized as mild (1–6 grades), moderate (7–12 grades), and severe level (13–18 grades).

### 2.5. Quantitative Real-Time Polymerase Chain Reaction (qRT-PCR)

Using TRIzol reagent (Invitrogen, Carlsbad, CA, USA), total RNAs were extracted from tissues and reversely transcribed to complementary deoxyribose nucleic acid (cDNA) using PrimeScript RT (TaKaRa, Tokyo, Japan). qRT-PCR was carried out using SYBR Green Kit (TaKaRa, Tokyo, Japan) with glyceraldehyde-3-phosphate dehydrogenase (GAPDH) as the internal reference. Primer sequences were shown in Table 1.

### 2.6. Statistical Analysis

Statistical product and service solutions (SPSS) 20.0 (IBM, Armonk, NY, USA) was used for statistical analysis. Data were expressed as *x̅* ± *s*. Differences between groups were compared by the *t*-test, and those among groups were compared by one-way ANOVA, followed by the SNK-q test. Prognostic and diagnostic potentials were assessed by Kaplan–Meier and ROC methods, respectively. Pearson's correlation test was applied for assessing the correlation between ALDH1 and other indexes. *P* < 0.05 was considered as statistically significant.

## 3. Results

### 3.1. Clinical Data of Subjects

In case group, there were 38 and 32 male and female patients, respectively, with an average age of 66.13 ± 2.69 years. Thirty-five males and thirty-five females were included in the control group with an average age of 65.9 ± 2.81 years. No significant differences in age and sex were identified between groups nor as history of hypertension, diabetes, dyslipidemia, coronary heart disease, and atrial fibrillation (*P* > 0.05, Table 2). It is concluded that baseline characteristics were comparable between the case and control groups.

### 3.2. Serum ALDH1 Level Increased in Acute Cerebral Infarction Patients

Compared with that of healthy volunteers, serum ALDH1 level was markedly higher in acute cerebral infarction patients (*P* < 0.05, Figure 1(a)), suggesting that the abnormally expressed serum ALDH1 level may be involved in the onset of cerebral infarction. ROC curves demonstrated that the area under curve (AUC) of ALDH1 in distinguishing acute cerebral infarction was 0.7912, with the sensitivity and specificity of 70% and 75.71% at the cut-off value of 1.5, respectively (*P* < 0.001, Figure 1(b)). It is proven that ALDH1 was a promising diagnostic marker in acute cerebral infarction. Moreover, 70 recruited patients were categorized to high-level group (*n* = 39) and low-level group (*n* = 31) by the median serum ALDH1 level. A worse survival was identified in high-level group, indicating that an increased serum ALDH1 level was unfavorable to the prognosis of cerebral infarction (HR = 1.521, *P*=0.0065, Figure 1(c)).

### 3.3. Neurological Deficits of MCAO Rats

To investigate the function of ALDH1 in acute cerebral infarction, MCAO model was performed, and 2 rats in cerebral infarction group died. Eighteen survivor rats presented neurological deficits, manifesting as circling to the right and unable to fully lift the right forepaw, suggesting the successful modeling of cerebral infarction. Rats in other two groups were all survived. mNSS was statistically significant among three groups (10.41 ± 2.15, 0.40 ± 0.09, and 0.45 ± 0.06 in cerebral infarction, sham operation, and control group, respectively) (*F* = 430.296, *P* < 0.001). However, no significant difference in mNSS was detected between sham operation and control groups (*P* > 0.05, Table 3).

### 3.4. Relative Levels of ALDH1, Smad2, Smad4, and p21 in Brain Tissues of MCAO Rats

Compared with those of sham operation and control groups, mRNA levels of ALDH1, Smad2, and Smad4 were markedly higher in cerebral infarction group, whilst p21 level was lower (*P* < 0.05). Their expression levels were similar between sham operation and control groups (*P* > 0.05, Figure 2).

### 3.5. Correlation between ALDH1 and mNSS, Smad2, Smad4, and p21

Interestingly, ALDH1 level in rat brain was positively correlated to mNSS of MCAO rats (*r* = 0.6182, Figure 3(a)) and relative levels of Smad2 and Smad4 (*r* = 0.7709 and 0.5335, *P* < 0.05, Figures 3(b) and 3(c)), which was negatively correlated to p21 level (*r* = 0.8207, *P* < 0.001, Figure 3(d)).

## 4. Discussion

With the aging population and improvement of life quality, cerebrovascular diseases, alongside cardiac diseases, and malignant tumors have become the top three causes of death. In China, at least 1.5 million people die of stroke annually, ranking 25% of all causes of death [15, 16]. Cerebral infarction is a common subtype of stroke that severely threatens human health and increases medical cost [15, 16].

ALDH1 is a zinc-containing enzyme located in the cytoplasm. It is responsible for catalyzing the oxidation of acetaldehyde to acetic acid. ALDH1 is expressed in hematopoietic and neural stem cells and is involved in cellular metabolism and stem cell differentiation. ALDH1 is a vital mediator of self-renewal and tumorigenesis of breast cancer cells [17]. In cervical cancer cells, highly expressed ALDH1 triggers proliferative, colony formation, and migratory capacities, serving as an independent risk factor for poor prognosis [18, 19]. Zheng and Zheng [20] suggested that cervical cancer cells overexpressing ALDH1 are featured by strong capacities of differentiation, self-renewal, and carcinogenesis. However, *in vivo* and *in vitro* cultured cervical cancer cells with a low abundance of ALDH1 lack these malignant phenotypes.

The novelty of the present study was that it is the first attempt for us to investigate the effects of ALDH1 on acute cerebral infarction and to explore the potential underlying molecular mechanism. Our results showed that serum ALDH1 level markedly increased in acute cerebral infarction patients. Its diagnostic and prognostic potentials in cerebral infarction were further verified. Through retrospectively analyzing follow-up data of recruited acute cerebral infarction patients, ALDH1 was found to be linked with 90-day all-cause mortality. Therefore, we believed that serum ALDH1 level was of significance in predicting adverse events and prognosis of acute cerebral infarction.

The Smad family directly participates in signal transduction of the transforming growth factor-beta (TGF-*β*) superfamily, which is critically important in regulating intracellular homeostasis and cell functions [21, 22]. A body injury triggers TGF-*β* release from cells, which binds cell surface receptors to induce a positive feedback to phosphorylate other TGF-*β* receptors. The Smad signaling is then activated by phosphorylated TGF-*β* receptors and further accelerates phosphorylation of intracellular Smad2 and Smad3, leading to a spatial conformational change [23, 24]. A heterotrimer complex formed by cross-linking with Smad4 is then translocated into nuclei, where mediates target gene transcription and induces inflammatory response, oxidative stress, and cell apoptosis [25]. Cyclin-dependent kinase inhibitor 1A (P21) is one of the targets of Smad4, which is associated with cell senescence, death, and apoptosis [26, 27]. In brain tissues of rats with acute cerebral infarction, we found that Smad2 and Smad4 were upregulated, and p21 was downregulated. ALDH1 level in brain tissues was positively correlated to mNSS, and relative levels of Smad2 and Smad4, but negatively correlated to p21 level. It is indicated that the influence of ALDH1 on neurological dysfunction caused by acute cerebral infarction may be attributed to the Smad signaling and its target gene p21.

## 5. Conclusions

Taken together, we have proven the clinical significance of serum ALDH1 level in predicting the onset of acute cerebral infarction and short-term poor prognosis. ALDH1 was closely linked to neurological dysfunction following cerebral infarction with the involvement of the Smad signaling and p21. Detection of serum ALDH1 level is simple and noninvasive, which is a promising method to be applied in monitoring cerebral infarction.

## Figures and Tables

**Figure 1:** Serum ALDH1 level increased in acute cerebral infarction patients. (a) Serum ALDH1 level in healthy volunteers and acute cerebral infarction patients; (b) ROC curves of ALDH1 in diagnosing acute cerebral infarction; (c) Kaplan–Meier curves of ALDH1 in predicting survival of acute cerebral infarction patients.

**Figure 2:** Relative levels of ALDH1, Smad2, Smad4, and p21 in brain tissues of MCAO rats.

**Figure 3:** Correlation between ALDH1 and mNSS (a), Smad2 (b), Smad4 (c), and p21 (d).

**Table 1:** Primer sequences.

Gene		Primer sequence
ALDH1 (Homo)	Forward	5′- GCCAGGTAGAAGAAGGAGATAAGGAGG -3′
	Reverse	5′- TATAATAGTCGCCCCCTCTCGGAAG -3′
ALDH1 (Rattus)	Forward	5′- GCCCTGGAGACGATGGATAC -3′
	Reverse	5′- TCCACTGCCAAGTCCAAGTC -3′
Smad2 (Rattus)	Forward	5′- TGGTGGTCGATAGTTTGTCCAT -3′
	Reverse	5′-GAACATAGACATAACCCTGAAGCTTTT-3′
Smad4 (Rattus)	Forward	5′- ACCAACTTCCCTAACTTTCCT -3′
	Reverse	5′- ACTATGGCTCGGTGCGAGAA -3′
p21 (Rattus)	Forward	5′- GAGAACTCGGGACCGCTTTC -3′
	Reverse	5′- TCCTGAGCGTGTTTGCTGTC -3′
GAPDH (Homo)	Forward	5′- ATCATCCCTGCCTCTACTGG -3′
	Reverse	5′- TGATGCTGGAGCTGGTAAAG -3′
GAPDH (Rattus)	Forward	5′- ATGGGGAAGGTGAAGG -3′
	Reverse	5′- TTACTCCTTGGAGGCC -3′

**Table 2:** Baseline clinical data between case and control groups.

Variable	Control group (*n* = 70)	Case group (*n* = 70)	t/*χ*^2^	*P*
Age (years)	65.9 ± 2.81	66.13 ± 2.69	1.437	0.153

Sex (n)				
Male	35	38	0.258	0.735
Female	35	32		

Hypertension (n)				
I.A.	23	28	0.771	0.483
N.A.	47	42		

Diabetes (n)				
I.A.	14	18	0.648	0.421
N.A.	56	52		

Dyslipidemia (n)				
I.A.	28	31	0.264	0.732
N.A.	42	39		

Coronary heart disease (n)				
I.A.	7	13	2.1	0.147
N.A.	63	57		

Atrial fibrillation (n)				
I.A.	4	6	0.431	0.512
N.A.	66	64		

I.A. is applicable; N.A. not applicable.

**Table 3:** mNSS scores in modeling rats.

Group	*n*	mNSS scores	*F*	*P*
Control	20	0.45 ± 0.06	430.296	<0.001
Sham operation	20	0.40 ± 0.09		
Cerebral infarction	18	10.41 ± 2.15 ^*∗*#^		

^*∗*^ *P* < 0.05 vs. control group; ^#^*P* < 0.05 vs. sham operation group.

## Data Availability

The datasets used and analyzed during the current study are available from the corresponding author upon reasonable request.

## References

[1] Zhou M., Wang H., Zhu J. (2016). Cause-specific mortality for 240 causes in China during 1990-2013: a systematic subnational analysis for the Global Burden of Disease Study 2013. *The Lancet*.

[2] Wang W., Jiang B., Sun H. (2017). Prevalence, incidence, and mortality of stroke in China. *Circulation*.

[3] Nadareishvili Z., Simpkins A. N., Hitomi E., Leigh D., Leigh R. (2019). Post-stroke blood-brain barrier disruption and poor functional outcome in patients receiving thrombolytic therapy. *Cerebrovascular Diseases*.

[4] Rabinstein A. A. (2020). Update on treatment of acute ischemic stroke. *Continuum*.

[5] Xiao D., Xiao Z. (2020). Pathophysiology and treatment of stroke: present status and future perspectives. *International Journal of Molecular Sciences*.

[6] Su Y., Qiu Q., Zhang X. (2010). Aldehyde dehydrogenase 1 A1-positive cell population is enriched in tumor-initiating cells and associated with progression of bladder cancer. *Cancer Epidemiology, Biomarkers & Prevention*.

[7] Ginestier C., Hur M. H., Charafe-Jauffret E. (2007). ALDH1 is a marker of normal and malignant human mammary stem cells and a predictor of poor clinical outcome. *Cell Stem Cell*.

[8] Tomita H., Tanaka K., Hara T., Hara A. (2016). Aldehyde dehydrogenase 1A1 in stem cells and cancer. *Oncotarget*.

[9] Holah N. S., Aiad H. A. E. S., Asaad N. Y., Elkhouly E. A., Lasheen A. G. (2017). Evaluation of the role of ALDH1 as cancer stem cell marker in colorectal carcinoma: an immunohistochemical study. *Journal of Clinical and Diagnostic Research*.

[10] Kang E. J., Jung H., Woo O. H. (2014). Association of aldehyde dehydrogenase 1 expression and biologically aggressive features in breast cancer. *Neoplasma*.

[11] Akinyemi R. O., Owolabi M. O., Ihara M. (2019). Stroke, cerebrovascular diseases and vascular cognitive impairment in Africa. *Brain Research Bulletin*.

[12] Suda S., Aoki J., Shimoyama T. (2018). Stroke-associated infection independently predicts 3-month poor functional outcome and mortality. *Journal of Neurology*.

[13] Shahjouei S., Cai P. Y., Ansari S. (2016). Middle cerebral artery occlusion model of stroke in rodents: a step-by-step approach. *Journal of vascular and interventional neurology*.

[14] Bieber M., Gronewold J., Scharf A. C. (2019). Validity and reliability of neurological scores in mice exposed to middle cerebral artery occlusion. *Stroke*.

[15] He J., Gu D., Wu X. (2005). Major causes of death among men and women in China. *New England Journal of Medicine*.

[16] Kim J., Song T. J., Park J. H. (2012). Different prognostic value of white blood cell subtypes in patients with acute cerebral infarction. *Atherosclerosis*.

[17] Neumeister V., Agarwal S., Bordeaux J., Camp R. L., Rimm D. L. (2010). In situ identification of putative cancer stem cells by multiplexing ALDH1, CD44, and cytokeratin identifies breast cancer patients with poor prognosis. *American Journal Of Pathology*.

[18] Rao Q. X., Yao T. T., Zhang B. Z. (2012). Expression and functional role of ALDH1 in cervical carcinoma cells. *Asian Pacific Journal of Cancer Prevention*.

[19] Yao T., Wu Z., Liu Y., Lin Q., Lin Z. (2014). Aldehyde dehydrogenase 1 (ALDH1) positivity correlates with poor prognosis in cervical cancer. *Journal of International Medical Research*.

[20] Zheng S. Y., Zheng P. S. (2013). High aldehyde dehydrogenase activity identifies cancer stem cells in human cervical cancer. *Oncotarget*.

[21] Khalil H., Kanisicak O., Prasad V. (2017). Fibroblast-specific TGF-*β*-Smad2/3 signaling underlies cardiac fibrosis. *Journal of Clinical Investigation*.

[22] Ruetz T., Pfisterer U., Di Stefano B. (2017). Constitutively active SMAD2/3 are broad-scope potentiators of transcription-factor-mediated cellular reprogramming. *Cell Stem Cell*.

[23] Wang L., Xu X., Cao Y. (2017). Activin/Smad2-induced histone H3 lys-27 trimethylation (H3K27me3) reduction is crucial to initiate mesendoderm differentiation of human embryonic stem cells. *Journal of Biological Chemistry*.

[24] Cortez V. S., Ulland T. K., Cervantes-Barragan L. (2017). SMAD4 impedes the conversion of NK cells into ILC1-like cells by curtailing non-canonical TGF-*β* signaling. *Nature Immunology*.

[25] Wu Y., Yu X., Yi X. (2017). Aberrant phosphorylation of SMAD4 thr277-mediated USP9x-SMAD4 interaction by free fatty acids promotes breast cancer metastasis. *Cancer Research*.

[26] Song W., Huang T., Yu L., Cheng Z. (2018). Expressions of DeltaNp63alpha, DPC4/Smad4 and P21 in cervical squamous cell carcinoma an their clinical significance. *Nan Fang Yi Ke Da Xue Xue Bao*.

[27] Cheng H., Chen C., Liu L. U., Li N. A., Li B. (2015). Expression of Smad4, TGF-*β*RII, and p21waf1 in esophageal squamous cell carcinoma tissue. *Oncology Letters*.

